The article "Design of a Smart Art Classroom System Based on Internet of Things" was published in 2022. Journal: Comput Intell Neurosci.

# Design of a Smart Art Classroom System Based on Internet of Things

**DOI:** 10.1155/2022/9257827

**Published:** 2022-04-12

**Authors:** Binbin Guo, Heung Kou, Yanbing Zhou

**Affiliations:** ^1^Department of Education, Graduate School of Sehan University, Yeongam-gun, Jeollanam-do 58447, Republic of Korea; ^2^Guangdong Medical University, Dongguan 523808, China

## Abstract

With the rapid development of the Internet of Things and to improve the teaching efficiency of the art classroom, a smart art classroom system based on the Internet of Things is proposed, which can effectively assist in teaching. First, we give the general design of the smart art classroom, including the composition of the hardware and software, and the construction method of the application system. Based on existing technologies such as RFID, smart camera, smart voice, smart terminal, and smart screen interaction, an all-around smart art classroom is constructed. Further, we present the design of an intelligent camera-based classroom assistance system based on face detection and facial expression recognition, which can effectively determine the status of students in class and can be used to assist in reminding teachers of their teaching tasks. Among them, face detection and facial expression recognition algorithms are designed based on different convolutional neural network architectures. Finally, experimental data sets are constructed to verify the accuracy of the used algorithms. The experimental results show that the detection accuracy of classroom faces is better than 95% and the accuracy of expression recognition is 88%, which can meet the application needs of intelligent art classrooms.

## 1. Introduction

In the past decades, with the rapid development of information technology, more and more network devices have been used in the classroom to assist in teaching. With the rapid development of the Internet of Things (IoT), IoT devices have been widely used in all walks of life [1–3]. Considering the needs of the classroom, a smart classroom system can be designed by combining IoT technology. Especially considering that the art classroom has a more significant demand for intelligent interaction and academic concentration judgment, the existing artificial intelligence and IoT technology can be combined to design an auxiliary teaching system, which can improve students' enthusiasm for learning on the one hand and assist teachers in judging the learning and studying status on the other.

Among the IoT technologies, radio frequency identification (RFID) [4] and IoT device networking [5] methods are developing rapidly, and different types of IoT devices can be connected in various ways to construct an internal network with barrierfree communication. Meanwhile, artificial intelligence technology has been developing rapidly in recent years, and technologies such as face detection [6] and facial expression recognition [7] based on images and semantic recognition have been developed rapidly, and a more intelligent classroom can be constructed by fully applying IoT-related technologies and artificial intelligence technologies. The design of a smart classroom helps to improve the efficiency of teaching and learning, especially in the art classroom, where it is highly significant to improve the level of service to students and the protection of important items within the art classroom.

Many researchers have tried to design different kinds of smart classrooms [8–10]. However, these types of smart classrooms do not have a more complete top-level design scheme, and they do not make enough use of the existing intelligent terminals and existing artificial intelligence methods. The hardware and software requirements are given, and a complete solution design is provided for constructing a more complete intelligent art classroom. Then, to make more effective use of artificial intelligence technology, this paper presents a classroom assistance system based on camera intelligence analysis and constructs face detection and expression recognition algorithms based on convolutional neural networks, which can effectively assist in analyzing and discriminating the status of students in the classroom. The experimental results show that the detection accuracy of classroom faces is better than 95% and the accuracy of expression recognition is 88%.

## 2. Overall Architecture Design of a Smart Art Classroom

A complete smart classroom system should include a variety of IoT devices, including cameras, microphones, audio, screens, RFID, projectors, computers, and other smart terminals. Different devices are connected together through the IoT network to form multiple functional subsystems, and through the functions and interactions of the subsystems, a complete intelligent classroom system is finally constructed.

The architecture of the intelligent art classroom is shown in Figure 1, and the system contains four subsystems, which are the intelligent monitoring system, intelligent voice system, intelligent identification system, and intelligent sensing system. The intelligent monitoring system mainly consists of networked cameras, which identify and analyze various targets and human behaviors through the intelligent image analysis technology of the cameras. The intelligent voice system consists of microphones and audio and uses voice recognition and analysis technology to assist in classroom teaching tasks. The main component of the smart tagging system is RFID, which includes RFID chips built into student cards and multiple devices in the classroom. The intelligent sensing system consists of a variety of sensors, including light, smoke, and fire sensors.

### 2.1. Intelligent Monitoring System

The architecture of the intelligent monitoring system is shown in Figure 2. The system mainly consists of multiple cameras, and the cameras are interconnected through a switch, cameras are configured with face detection [11], face recognition [12], facial expression recognition [13], fall detection [14], fight detection and other functions. To carry out a comprehensive analysis of the detection results of multiple cameras, an analysis device is always equipped. The analysis device can be a server or a small terminal device, taking into account the installation environment inside the classroom, which is usually equipped with a small intelligent analysis box. Of course, some intelligent classrooms will also be equipped with a unified server in the server room, for the synthesis of the analysis results of all the classroom cameras in the school.

Smart cameras usually have the following functions:

1. Face detection: used to detect the face of each student in the course for subsequent face recognition and expression analysis.
2. Face recognition: identifies each student in the classroom and is used to analyze and record the performance of each student.
3. Expression recognition: through the analysis of students' posture and expressions, students' concentration can be analyzed, which can be used to assist teachers in analyzing the effect of lectures so as to adjust the lecture content and teaching methods.
4. Fall detection: it is mainly used to detect accidental falls during students' activities in class, mainly based on the detection of human targets and joint point analysis to discriminate and can provide a timely warning when a fall is detected to improve classroom safety.
5. Fight detection: mainly for the detection of classroom fights, when a fight is detected, it will automatically send relevant alarm information to the teacher's cell phone to improve classroom safety.

Intelligent analysis devices can be designed using embedded intelligent chips. For example, you can use Huawei Hisilicon SOC, Qualcomm Snapdragon SOC, or Nvidia Jetson SOC. These SOCs usually contain powerful hardware decoding chips and artificial intelligence inference chips, which can support the decoding of multiple camera video and real-time intelligent analysis, and the cost of such chips is much lower than the server, which can effectively improve the cost performance of the system.

Computer vision is the current hot technology in artificial intelligence and constructing an intelligent surveillance system can make use of current advanced computer vision technology to effectively improve the intelligence of the system [15]. To this end, this paper constructs an intelligent monitoring system based on Internet of Things technology and artificial intelligence technology, which can effectively improve classroom efficiency and security.

### 2.2. Intelligent Voice System

The architecture of the intelligent voice system is shown in Figure 3. The system mainly consists of a microphone, speech recognition system, and audio. Among them, the microphone is an input device, which is used to collect speech information in the classroom. The speech recognition system recognizes the collected speech and understands the semantics, makes decisions and selects the best solution through the semantics, and finally converts it into speech output to the audio for the reply. With the interactive semantic recognition function, the IoT devices in the classroom can be jointly controlled by voices to improve classroom efficiency.

In a semantic recognition system, the first step is to recognize the voices as text [16] that can be processed by the computer. The text is then divided into words, and further semantic analysis and understanding [17] are performed. Semantic analysis and understanding require the application of deep neural networks, which have also been a hot research area in deep learning in the past few years. On the basis of semantic understanding, it is necessary to select the appropriate reply message, and usually, a question and answer system needs to be constructed, through which the decision is made and the best reply solution is given. In the smart classroom, the speech recognition system can be linked with a variety of IoT devices, and the actions of the devices can be controlled by voice to achieve more efficient classroom interaction.

In the intelligent IoT system, the linkage function between devices based on speech recognition system has become more and more mature, and the devices are associated and controlled through a unified speech recognition terminal, which has been maturely applied in the home IoT system. In the smart classroom, since there are still few IoT devices and the way of linkage between devices is still unclear, it is necessary to study the way of linkage combination of speech recognition and control for existing classroom IoT devices to construct a more intelligent classroom system.

### 2.3. Intelligent Identification System

RFID is a wireless communication technology that can be used to construct electronic tags without having to manually read them. Wireless technology is used to achieve automatic reading and management of tags. RFID is a common technology in the IoT [18]. It is always used in intelligent storage management [19] for intelligent classroom systems. RFID can be used to construct an asset management system, implant RFID on the equipment used in the classroom, and carry out intelligent management of assets entering and leaving the classroom. The framework is shown in Figure 4. The main areas include the following:

1. *Statistics on the entry and exit of assets such as tables and chairs.* Tables and chairs are the most basic asset facilities in the classroom. Now that the tables and chairs are becoming more and more functional and valuable, implanting RFID can effectively prevent the theft of tables and chairs. Through the tables and chairs in and out of the classroom, the door implanted induction equipment to generate access records is combined with the access time and the number of students in the current classroom teacher. If registered students or teachers are not found in the classroom during the movement of tables and chairs, it is timely to generate alarm information and send it to the management.
2. *Management of student identity.* RFID chips are implanted in the student cards, which generate records when students enter and leave the classroom and can be used for attendance or analysis of abnormal events.
3. *Management of painting equipment.* A smart art classroom can be equipped with more intelligent painting equipment. In order to achieve the safe management of painting equipment, RFID chips can be implanted in the equipment. Each time the equipment is in and out of the classroom will generate records. And it can be bound with the record of a student card to determine whether it is brought out by students so that the belonging status of the equipment can be accurately tracked.
4. *Management of other equipment.* Smart art classrooms have added many IoT devices. In these devices, implanted RFID chips can effectively achieve the management of assets.

With RFID technology, we can achieve real-time asset attribution status of the smart art classroom for recording and management, with the real-time display of the classroom screen, to achieve a more intelligent equipment management system to assist the school's asset management.

### 2.4. Intelligent Sensing System

The purpose of the intelligent sensing system is to create an intelligent, comfortable, and safe classroom scene based on multiple types of sensors [20]. From the perspective of intelligence and comfort, human sensors, light sensors, and smart lights can be combined to achieve adaptive adjustment of light brightness in the classroom and achieve a more comfortable classroom environment. Considering that there are more electrical devices in the classroom, the security aspect also needs to be strengthened. For example, a smoke alarm, temperature sensor, and odor alarm can be equipped to detect the occurrence of fire and set off an alarm immediately. The framework is shown in Figure 5. Specific construction measures are as follows:

1. *Construct a comfortable classroom environment based on multiple sensors.* Using human sensors to sense the teachers or students entering and leaving the door, start the lights in the classroom and turn on the air conditioner when the first student enters the classroom, and sense the outdoor temperature through the temperature sensor so as to automatically adjust the air conditioning temperature as well as the cooling and heating modes. The indoor light is sensed in real-time and adjusted to the right brightness by the smart light. After all the students leave the classroom, all lights and devices are turned off and enter hibernation mode, waiting for the next wake-up call.
2. *Construct a safe classroom environment based on multiple sensors.* As there are more electrical devices in the classroom, to prevent fires in the classroom, smoke alarms and odor sensors can be equipped in multiple directions in the classroom to start fire extinguishing devices and alarm in time when smoke or larger odors are generated by any device.

Various types of sensors are inaccessible components of the IoT system, and a more intelligent and comfortable IoT application scenario can be constructed based on various sensing devices. With the intelligent sensing system constructed in this paper, we can provide a more comfortable and safe environment for the intelligent art classroom students. Limited by the space of this paper, more intelligent application scenarios cannot be described. Sensors can also be linked with intelligent voice, intelligent monitoring, and other systems to create a more intelligent application scenario together.

## 3. Face Detection and Expression Recognition in Intelligent Monitoring Systems

In order to achieve a more intelligent surveillance system, face detection and facial expression recognition algorithms are necessary. To this end, this paper designs a face detection algorithm and a facial expression recognition algorithm to provide an algorithmic basis for an intelligent surveillance system.

### 3.1. Face Detection Algorithm

The purpose of the face detection algorithm is to find out where a face is located from an image and to give a localization of the key points of the face. Although the structure of a human face is determined, consisting of parts such as eyebrows, eyes, nose, and mouth, it is approximately the same as a rigid body. Due to the changes in posture and expression, the appearance differences of different people, illumination, and occlusion, it is difficult to accurately detect human faces under various conditions. The main key problems with face detection are as follows: faces can appear at any position in the image; faces exist in different sizes; faces exist in different poses and perspectives in the image; faces are easily occluded. Because the face may appear anywhere in the image, a fixed-size window is used in the detection process to scan the image from top to bottom and from left to right to determine whether the subimage in the window is a face, which is called sliding window technology. To detect different sizes of faces in the images, the image pyramid is also constructed by scaling up or down the image, and each scaled image is scanned using the above method. Due to the use of sliding window scanning technology, where the image is repeatedly scaled and scanned, the whole detection process will be very time-consuming.

The previous best detectors can be roughly divided into two categories: the first category is mainly based on the RPN network and adopts the two-stage detection mechanism. After end-to-end training, RPN generates high-quality regional suggestions for further use in the faster RCNN [21]. The other class is based on a single-stage single point detector (SSD), which discards the RPN to directly predict the box and confidence. Currently, single-stage face detection frameworks are more concerned with higher inference efficiency and direct system deployment.

Early work on face detection relied heavily on hand-designed features, such as Haar features, control point settings, and edge direction histograms. However, the hand-designed features lacked guidance. With the development of deep neural networks, the features of manual design have been replaced by convolutional neural networks. For example, cascaded RCNN and MTCNN use CNN as a sliding window detector in the image pyramid to construct the feature pyramid. However, using image pyramids is very slow and out of memory. Therefore, most two-stage detectors extract features on a single scale. RCNN obtains region suggestions through a selective search algorithm and then classifies each standardized image region through CNN forwarding. The RPN network is used by faster RCNN and RFCN to generate original area recommendations. In addition, to extract features from each region, location-sensitive POI pooling and ROI pooling can be used.

Recently, some studies have shown that multiscale feature maps perform better for tutorials of small targets, in particular, SSD, MS-CNN, SSH, and S3FD predicting boxes on multiple feature layers. It fuses multilayer features for segmentation. Although FPN segmentation style networks similar to PyramidBox achieve good results, they do not consider the information of the current layer. Unlike the above approaches that ignore the contextual information between anchors, a feature enhancement module containing multiple layers of expanded convolutional layers is used to enhance the semantics of features. The architecture of the face feature extraction network is shown in Figure 6.

The network structure uses VGG16 as the backbone. The feature enhancement module first samples the higher-level feature maps and multiplies them at the element level with the current layer. Finally, slice the feature map into three parts, followed by three subnetworks containing different numbers of null convolution layers. The details are shown in Figure 7.

The convolution can be expressed by

(1) $$\begin{array}{c} \left\{\begin{array}{c} r_{i}=f\left(w\cdot X+b\right),\\ X=\left[x_{i},x_{i+1},...,x_{i+h}\right], \end{array}\right. \end{array}$$

where *r*_*i*_ indicates the convolution result, *f* is the nonlinear activation function, *w* is the parameters of the convolution filter, *b* is the bias term, *X* is the input vector of a window, and *h* is the kernel size of convolution.

Dilation convolution achieves alternate convolution and increases the perceptual field while maintaining image resolution. Assuming that the convolution kernel size of the hole convolution is *k* and the hole size is *d*, the perceptual field is calculated as follows:

(2) $$\begin{array}{c} \left\{\begin{array}{c} k{}^{\prime }=k+\left(k-1\right)\times \left(d-1\right),\\ R_{i+1}=R_{i}+\left(k{}^{\prime }-1\right)\times S_{i}, \end{array}\right. \end{array}$$

where *R*_*i*_ denotes the perceptual field and *S*_*i*_ denotes the product of the step lengths of all layers before this layer.

The feature enhancement module utilizes feature map upsampling and null convolution to extract features, which are finally stitched together into a new feature map that can be described as follows:

(3) $$\begin{array}{c} \left\{\begin{array}{c} E_{c}=f_{\text{concat}}\left(f_{\text{dilation}}\left(N_{c}\right)\right),\\ N_{c}=f_{\text{prod}}\left(O_{c},f_{\text{up}}\left(O_{c}\right)\right), \end{array}\right. \end{array}$$

where *E*_*c*_ denotes the enhanced features, *f* denotes the operations, *O*_*c*_ denotes the original cells, and *N*_*c*_ denotes the nonlocal neuron cells.

The usual detection target loss is a weighted summation of classification and regression. Smoothed L1 loss can be used to stop the gradient explosion, while class imbalance is the main reason for performance, and dynamically scaled cross-entropy can be used. RepLoss can be used for pedestrian detection, which improves the performance of occluded scenes. FANet proposes hierarchical feature pyramids and hierarchical losses. However, the proportion of anchors used in FANet remains the same in different phases. In this paper, different anchor sizes at different stages are chosen to simplify the features. We used to multitask loss because it simplifies the training task for both the original and augmented feature maps in two ways. The anchor-based multitask loss function is defined as follows:

(4) $$\begin{array}{c} L_{S}=\frac{1}{N_{c}}\left(\sum_{i}L_{c}+\frac{\beta }{N_{l}}\sum_{i}p_{i}L_{l}\right). \end{array}$$

Compared with the enhanced feature map at the same layer, the original feature map has less information available for classification but has higher resolution information. The higher resolution facilitates the detection and classification of small faces when the original feature map can be used. Therefore, the multitask loss function for smaller anchors is defined as follows:

(5) $$\begin{array}{c} L_{F}=\frac{1}{N_{c}}\sum_{i}L_{c}+\frac{\beta }{N_{l}}\sum_{i}p_{i}L_{l}. \end{array}$$

The losses of the two layers can be weighted and summed to obtain the entire asymptotic anchor loss, which is defined as follows:

(6) $$\begin{array}{c} L_{p}=L_{F}+\lambda L_{s}. \end{array}$$

The main idea of progressive anchor loss (PAL) is that not only is the anchor size on different levels of special different, but also the anchor size on the original feature and the enhanced special on the same level is different. Using PAL can effectively improve the accuracy of anchors.

### 3.2. Facial Expression Recognition Algorithm

Over the past few decades, many researchers have made more significant progress in facial expression recognition (FER) by studying a large number of face expression datasets collected in different scenarios. A typical facial expression recognition (FER) system usually consists of three phases, face detection, feature extraction, and facial expression recognition. In the face detection phase, there have been many advanced results in face detection that can be used for face localization and detection in complex real-life scenes. The detected faces are then transformed and aligned. For feature extraction, researchers have devised various methods to extract facial geometry and facial expression change features. The early features are mainly based on artificially designed features, such as texture-based local features, geometry-based overall features, and hybrid features. Among them, the texture-based features mainly include HOG, LBP histogram, Gabor wavelet coefficients, SIFT, etc. The geometry-based global features are mainly based on five-sense positions and surrounding boundary marker points. Hybrid features combine a variety of image texture features and ensemble features, which can further enrich the characterization ability of features. In recent years, various CNNs have been mainly used to automatically extract facial features from human faces. The accuracy of the face detection algorithm has a large impact on the accuracy of expression recognition. For this reason, based on the face detection algorithm in the previous subsection, an expression recognition algorithm is introduced in this subsection.

For the large-scale FER datasets collected from public channels, the quality of the collected images cannot be guaranteed due to the limitations of the acquisition conditions, and the annotation of low-quality images in the annotation process is easily influenced by the subjectivity of the annotators, so there are a large number of low-quality annotations in the existing large-scale FER datasets. Typically, an uncertain sample in the dataset may have the following effects on the training of FER: first, it may lead to overfitting of the model to a small number of mislabeled, low-quality samples. Second, the mislabeled samples can affect the convergence of the model and prevent the best training results. Third, a high percentage of mislabeled samples can make the model illogical in the early stages of optimization.

To solve these problems, a simple but effective method called self-cure network (SCN) is used to suppress the uncertainty of large-scale facial expression recognition. The SCN contains three key modules: self-attention weighting, rank regularization, and noise relabeling. Facial features are first extracted using a backbone CNN. Then, the weighting module based on the self-attention mechanism automatically generates the weight information of each image through the network. The training weights of incorrectly labeled images are reduced by self-learning the weight information through the weight loss function. The rank regularization module ensures that important features are learned in the feature map area module and achieves suppression of erroneous samples by different weight information. The last module is the relabeling module, and this module improves the data accuracy by comparing the maximum prediction probability and relabeling the low-quality samples. The architecture is shown in Figure 8.

Given a batch of images, the face features are first extracted using a backbone CNN. Then, the weighting module based on the self-attentive mechanism learns the weights of each image by iterative training and calculates the weighting of importance for the samples. Low-quality images are assigned lower weights. The images are then reordered by weight and divided into two groups using the ranking regularization module, and regularization is achieved by calculating and balancing the difference between the average weights of the two groups. The rank regularization module ensures that the feature extraction module learns some more important features in the beginning stage, focusing on typical samples and suppressing low-quality samples.

The weighting module based on the attention mechanism is mainly used to calculate the importance weights of different quality samples and perform the weighting calculation during the training process. It ensures that high-quality samples can get better weights and low-quality samples get lower weights, thus improving the effectiveness of feature learning. The weights are calculated as follows:

(7) $$\begin{array}{c} \alpha_{i}=\sigma \left(W^{T}x_{i}\right), \end{array}$$

where *α*_*i*_ denotes the output weight, *x*_*i*_ is the input, *W* is the inner parameter, and*σ* is the sigmoid activation function.

With attention weights, loss weighting can be performed. The logarithmic weighting method was chosen in this paper. The logarithmically weighted cross-entropy loss (WCE-Loss) formula is

(8) $$\begin{array}{c} L_{W}=-\frac{1}{N}\sum_{i=1}^{N}\log\frac{e^{\alpha_{i}}W^{T}x_{i}}{\sum_{j=1}^{C}e^{\alpha_{i}}W_{j}{}^{T}x_{i}}. \end{array}$$

In the weighting module based on the self-attentive mechanism, the weight values of the samples are taken in the range [0, 1], and the weight values of all samples are normalized using the rank regularization module. In the rank regularization module, the attention weights obtained from training are sorted in descending order and divided into two groups for processing, and the weight values between the two groups are compared and balanced. The formula for the rank regularization loss (RR-Loss) is shown as follows:

(9) $$\begin{array}{c} L_{RR}=\max\left\{\text{0},\delta_{1}-\left(\alpha_{H}-\alpha_{L}\right)\right\}, \end{array}$$

where *α*_*H*_ and *α*_*L*_ can be defined as

(10) $$\begin{array}{c} \alpha_{H}=\frac{1}{M}\sum_{i=0}^{M}\alpha_{i},\\ \alpha_{L}=\frac{1}{N-M}\sum_{i=M}^{N}\alpha_{i}. \end{array}$$

The final weighted loss function is as follows:

(11) $$\begin{array}{c} L_{a}=\gamma L_{RR}+\left(1-\gamma \right)L_{W}. \end{array}$$

For each sample, the maximum prediction probability is compared with the probability of a given label. If the maximum prediction probability is higher than one of the given labels with a threshold value, the sample is assigned to a new pseudolabel. The formula for the relabeling module is described as follows:

(12) $$\begin{array}{c} y{}^{\prime }=\left\{\begin{array}{c} l_{\text{max}},\text{if }P_{\text{max}}-P_{gt}>\delta_{2},\\ l_{\text{org}},\text{otherwise.} \end{array}\right. \end{array}$$

SCN can effectively enhance the suppression effect on unclear samples by weight calculation and relabeling of samples, thus improving the accuracy of expression recognition.

## 4. Experiments and Results Analysis

In this paper, three experiments are designed to analyze the accuracy of the face detection algorithm, the accuracy of face expression recognition, and the computational speed of the AI-based chip.

### 4.1. Face Detection Experiment

In this experiment, the face detection algorithm is trained and tested using the Wider Face dataset, a publicly available dataset of faces collected in multiple environments, which can effectively verify the accuracy of the facial recognition algorithm. In order to verify the accuracy of the face detection algorithm, a public dataset called Wider Face is used to train and test the algorithm in this paper. To verify the accuracy of the facial expression recognition algorithm, the algorithm is trained and tested using the public dataset RAF-DB.

The face detection algorithm training loss curve is shown in Figure 9. The ROC curve is shown in Figure 10. The training results show that the face detection algorithm can achieve good convergence and can achieve an effective detection effect.

To verify the effectiveness of the improved anchor matching algorithm, a comparison experiment was conducted with the traditional anchor matching algorithm on different sizes of face scales, and the results are shown in Figure 11. The comparison results show that the improved anchor matching algorithm works significantly better than the traditional algorithm on multiple sizes of face scales.

We tested the face detection algorithm on the test set of Wider Face and tested the detection accuracy on three datasets: hard, medium, and easy. The best results were 10 times as shown in Figure 12. The results show that the face detection algorithm has an accuracy of over 95% on the easy dataset and 90% on the hard dataset, which can meet the face detection needs in the smart art classroom.

### 4.2. Facial Expression Recognition Experiment

In order to verify the accuracy of the facial expression recognition algorithm, this paper conducted training and testing using the publicly available dataset RAF-DB, which is a real-world collection of face expressions in multiple scenes with certain representativeness. The training loss curve and ROC curve of this experiment are shown in Figures 13 and 14. The training results show that the facial expression recognition algorithm can achieve good convergence and can achieve an effective detection effect.

We tested the face detection algorithm on the test set of RAF-DB. The best results were 10 times as shown in Figure 15. The results show that the face detection algorithm has an accuracy of over 88%, which can meet the face detection needs in the smart art classroom.

## 5. Conclusion

This paper gives a scheme of a smart art classroom system that contains four subsystems, namely, an intelligent monitoring system, an intelligent semantic system, an intelligent tagging system, and an intelligent sensing system. Among them, the intelligent monitoring system is mainly composed of camera networking, which constitutes the function of identifying and analyzing the behavior of various targets and people through the intelligent image analysis technology of the camera. The intelligent voice system mainly has a microphone and audio networking composition, through the background of voice recognition and analysis technology, to assist the teacher with classroom teaching tasks. The smart tagging system mainly consists of RFID, which can construct a reliable tagging network through RFID chips built into student cards and multiple devices in the classroom. The intelligent sensing system consists of a variety of sensors, including light, smoke, fire, and other sensors, which can effectively improve classroom safety and comfort. Meanwhile, a face detection algorithm and a facial expression recognition algorithm are analyzed and validated on public datasets. The experimental results show that the face detection algorithm and expression recognition algorithm can achieve high detection accuracy and can meet the application requirements of the smart art classroom.

## Figures and Tables

**Figure 1:** Architecture of smart art classroom.

**Figure 2:** Architecture of intelligent monitoring system.

**Figure 3:** Architecture of intelligent voice system.

**Figure 4:** Architecture of intelligent identification system.

**Figure 5:** Architecture of intelligent sensing system.

**Figure 6:** Architecture of face feature extraction network.

**Figure 7:** Architecture of feature enhancement module.

**Figure 8:** Architecture of SCN.

**Figure 9:** Training loss curve of the face detection model.

**Figure 10:** ROC curve of the face detection model.

**Figure 11:** Comparison results of the improved and traditional anchor matching algorithms.

**Figure 12:** Detection accuracies on the easy, medium, and hard datasets.

**Figure 13:** Training loss curve of the facial expression recognition model.

**Figure 14:** ROC curve of the facial expression recognition model.

**Figure 15:** Detection accuracies on the RAF-DB datasets.

## Data Availability

The data used to support the findings of this study are available from the corresponding author upon request.
